# Superior efficacy of the antifungal agent ciclopirox olamine over gemcitabine in pancreatic cancer models

**DOI:** 10.18632/oncotarget.23164

**Published:** 2017-12-08

**Authors:** Chrysovalantou Mihailidou, Pavlos Papakotoulas, Athanasios G. Papavassiliou, Michalis V. Karamouzis

**Affiliations:** ^1^ Molecular Oncology Unit, Department of Biological Chemistry, Medical School, National and Kapodistrian University of Athens, 11527 Athens, Greece; ^2^ 2^nd^ Department of Medical Oncology, Theagenion Hospital, 54007 Thessaloniki, Greece; ^3^ First Department of Internal Medicine, Laiko Hospital, Medical School, National and Kapodistrian University of Athens, 11527 Athens, Greece

**Keywords:** pancreatic cancer, ciclopirox olamine, pharmacodynamic activity, gemcitabine, human pancreatic tumor xenograft models

## Abstract

Ciclopirox olamine (CPX) is an antifungal agent that has recently demonstrated promising anti-neoplastic activity against hematologic and solid tumors. Here, we evaluated CPX compared with gemcitabine alone as well as their combination in human pancreatic cancer cell lines; BxPC-3, Panc-1, and MIA PaCa-2 and in humanized xenograft mouse models. We also examined the preclinical pharmacodynamic activity of CPX. CPX caused a pronounced decrease in cell proliferation and clonogenic growth potential. These inhibitory effects were accompanied by induction of reactive oxygen species (ROS), which were strongly associated with reduced Bcl-xL and survivin levels and activation of a panel of caspases, especially caspase-3, and finally resulted in apoptotic death. CPX-induced apoptosis was associated with reduced pEGFR (Y1068) and pAkt (Ser473) protein levels. Additionally, decreased proliferation was observed in CPX-treated xenografts tumors, demonstrating unique tumor regression and a profound survival benefit. Finally, we showed that CPX significantly abrogated gemcitabine-induced ROS levels in pancreatic tissues. These pre-clinical results have verified the superior antitumor efficacy of CPX over gemcitabine alone, while their combination is even more effective, providing the rationale for further clinical testing of CPX plus gemcitabine in pancreatic cancer patients.

## INTRODUCTION

Pancreatic cancer is the third most frequent cause of cancer-related death in both women and men, with a rather low five-year survival rate [1]. The majority of pancreatic cancers are ductal adenocarcinomas that completely mimic infiltrative neoplasm and present early metastatic dissemination to distant target organs [2]. Currently, pancreatectomy is the only curative treatment option for localized pancreatic cancer [3]. However, this disease is usually diagnosed at an advanced stage and most available treatments finally render ineffective, portending to dismal survival [4, 5]. *KRAS* is mutated in approximately 95% of advanced and/or metastatic pancreatic carcinomas and is a well-confirmed driver of pancreatic tumor growth and progression. However, in spite of many efforts, an efficient anti-RAS agent, till now, has not reached the clinic [6]. Pancreatic cancer is characterized by a desmoplastic stroma that can encompass 70%–80% of the tumor volume. Consequently, the delivery of drugs to the pancreatic tissue is low and the tumor pancreatic tissue is characterized by low bioavailability [6]. Hence, more research is required with novel therapeutic strategies that may overcome the pathophysiological obstacles of this life-threatening malignancy.

Gemcitabine is an antimetabolite and among the most frequently prescribed anticancer agents worldwide. It is a nucleoside analog which must be converted into active mono-, di-, or tri-phosphorylated nucleotides to exert its full antitumor action either by targeting ribonucleotide reductase or through inhibition of DNA synthesis [7]. For years, gemcitabine single-agent has been the first-line chemotherapy option for treating locally advanced and/or metastatic pancreatic carcinomas [8]. Recent data have indicated a modest survival advantage when gemcitabine is combined with nab-paclitaxel [9]. However, this combination exhibited higher toxicity compared to gemcitabine alone. Therefore, treatment with gemcitabine alone is still considered the mainstay care drug and is usually the backbone on which new agents are pre-clinically and clinically evaluated [10]. However, gemcitabine chemotherapy provides only modest improvements in long-term and/or disease-free survival [11]. Therefore, other agents or drug combinations need to be assessed to circumvent tumor resistance in this challenging malignancy.

Ciclopirox olamine (CPX) is a synthetic antifungal broad-spectrum agent used against bacterial infections over the last decades [12–14]. CPX agent is a well-recognized iron chelator, which inactivates the action of the iron-containing enzymes in a variety of tissues and organisms with pathological situations [15], contributing to cell death either via over-production of ROS or via mediators of ROS that are related to cell death [16]. This is indicated as the most important mechanism of CPX's action [17]. Moreover, mechanistic studies showed that, besides the effects of iron, CPX inhibits nucleotide-binding proteins [18] and mTOR (mammalian target of rapamycin) signaling and also promotes autophagy in immune and mammalian cells [19]. Further studies showed that CPX chelation inhibits Wnt signaling and cell growth [20–22] and simultaneously suppresses survivin, which is involved in pro-survival signaling [21, 23].

Moreover, CPX has been recently identified to possess antitumor activity in several preclinical cancer models, such as breast carcinoma, rhabdomyosarcoma, colon adenocarcinoma [23] and hematological malignancies, such as multiple myeloma and acute leukemia [24–26]. A recent research revealed that CPX promoted apoptosis in AML (Acute Myeloid Leukemia) cells and suppressed engraftment of primary AML cells in NOD/SCID mice without evidence of organ toxicity or body weight loss [24]. A study conducted by Zhou and his group showed that CPX diminished Cyclin A, B1, D1, E, CDK2 (cyclin-dependent kinase 2), CDK4 (cyclin-dependent kinase 4), Bcl-xL and survivin, protein levels and enhanced CDK inhibitor p21 (Cip1) and Bcl-2 cleavages, protein levels [23]. Moreover, CPX has lately been reported to synergize with parthenolide to further enhance anti-leukemic activity. The combination of both drugs demonstrated mTOR inhibitory activity by activating autophagy in mammalian cells [26].

The rapid approval of CPX for topically treatment against strong fungicidal effects is supported by metabolic, pharmacokinetics, pharmacodynamics, clinical and toxicological data. CPX is nowadays administered topically. However, due to the repositioning of CPX as a potential therapeutic agent for treatment of patients with hematologic cancers [27, 24], systemic administration of this agent has been intensively evaluated [24]. Older studies confirmed that oral administration of CPX in mice, rabbits, and rats at dose levels ranging from 1700 to 3290 mg/kg did not show any systemic toxic effects [28, 29]. Also, repeated administration of CPX at 10μM was tolerable to dogs and rats without toxicity [29]. Additionally, animal studies [23, 24, 27, 29] and an employed human oral dosing study [25], suggest that CPX drug safety is satisfactory for human clinical trials [25]. Keller and his group showed that after oral administration of radiolabeled CPX to humans, 96% of the administered CPX was recovered from urine [29]. This research group verified that drug concentrations of CPX appeared pharmacologically achievable, although it's half-life is short and requires dosing several times a day. They noticed, however, that the drug seemed to be well absorbed [29]. Minden and his research group [25] conducted the first-in-human phase I clinical trial (NCT00990587) for the treatment of advanced hematologic malignancies. They showed that CPX (oral administration) at a dose of 40 mg/m^2^ for 5 days (per cycle) is well tolerated in all patients without any major toxicity. In addition, disease stabilization was reported, allowing for this group of patients to get additional cycles of treatment. An hematologic improvement was recorded in two-thirds of the 23 patients receiving study treatment, supporting a superior therapeutic index of CPX [25]. Suppression of survivin expression in PBMCs (peripheral blood mononuclear cells) isolated from refractory hematologic cancer patients, was noticed following the once-daily CPX treatment at doses higher than 10 mg/m^2^, indicating biological and pharmacodynamic activity of this repositioned drug. Gastrointestinal toxicity was only reported in patients receiving the highest dose (80mg/m^2^) administered with higher frequency (four times per day), but not at lower doses or at a less frequent dosing schedule [25].

Taken into consideration all the aforementioned, in this study, we evaluated the efficacy of CPX compared with gemcitabine alone as well as their combination in pancreatic tumor models. The choice of CPX was driven by CPX's mechanism of action through general iron chelation. We have demonstrated a superior anti-tumor activity of CPX over gemcitabine alone, while their combination was even more effective.

## RESULTS

### CPX potentiates chemosensitivity and triggered a more pronounced decrease in cell proliferation over gemcitabine treatment in various human pancreatic cell lines

To determine the sensitivity of CPX we chose the BxPC-3, PANC- 1 and MIA-PaCa-2. These cell lines are derived from primary tumors with moderate-to-poorly differentiation and with differential mutational status of KRAS (wild type for BxPC-3; mutant for PANC- 1, MIA-PaCa-2), CDKN2A/p16, TP53 and SMAD4/DPC4 [31]. Initially, we investigated the sensitivity of BxPC-3, PANC- 1 and MIA-PaCa-2, to gemcitabine employing the cell viability assay, the MTT assay. Firstly, cells were exposed for 72 hours to gradually increasing gemcitabine concentrations (0–100 mM). MIA-PaCa-2 cells demonstrated the greater sensitivity to gemcitabine with an IC_50_ (half maximal inhibitory concentration) at a concentration equal to 0.1mM. BxPC-3cells exhibited mildly sensitivity with an IC_50_ equal to 10mM. PANC- 1 cells showed to be the most resistant and hold the highest IC_50_ at a concentration higher than 50mM (Figure 1A). BxPC-3, PANC- 1, and MIA-PaCa-2 were also cultured for 72 hours with gradually increasing CPX concentrations (0–20 μM) (Figure 1B, 1D). Once more, MIA-PaCa-2 cells demonstrated the greater sensitivity to CPX with an IC_50_ at concentration 0.5μM. BxPC-3cells cells also exhibited modest sensitivity with an IC_50_ at a concentration equal to 1 μΜ (Figure 1B). PANC- 1 cells acquired sensitivity with an IC_50_ at a concentration equal to 5 μΜ (Figure 1B). Treatment with gemcitabine (10 mM) alone or CPX (5 μM) alone for 72 h reduced cell proliferation of BxPC3, PANC-1 and MIA PaCa-2 cells in a concentration-dependent manner, that differs between the cell lines, as shown in Figure 1A and 1B. CPX and gemcitabine inhibited cell proliferation of human pancreatic cells in a dose-dependent manner but with differential responses. Most obvious CPX triggered a more uniform suppression of proliferation than gemcitabine treatment. To investigate the improvement of gemcitabine antitumor effect by CPX combination strategy, cells were exposed to gemcitabine co-cultured with CPX (Figure 1C). BxPc3, Panc1 and MIA PaCa-2 cells were highly susceptible to respond to the combined strategy (Figure 1C). This experiment proposes higher *in vitro* cytotoxic activity of CPX and gemcitabine compared with CPX alone or gemcitabine alone. This MTT assay pointed that CPX augmented gemcitabine sensitivity of these three pancreatic cell lines.

**Figure 1:** CPX showed higher inhibitory effects on cell proliferation and colony forming ability as well as further stimulation of the ROS generation compared to gemcitabine treatment, in human pancreatic cell lines BxPC-3, PANC-1 and MIA-PaCa-2 cells were incubated with a range of (**A**) CPX increasing doses (0 −20 μM) and (**B**) Gemcitabine increasing doses (0 – 100 mM). Next, cell viability was analyzed using colorimetric MTT metabolic activity assay. (**C**) Cells were exposed to gemcitabine co-incubated with CPX, at concentration 10 mM and 5 μM respectively, and were analyzed using colorimetric MTT metabolic activity assay. (**D**) Chemical structure of CPX (ciclopirox olamine). (**E**) Clonogenic survival of BxPC-3, PANC-1 and MIA-PaCa-2 following exposure to gemcitabine (10 mM) and CPX (5 μM) singly or in combination. Results are expressed as percentages vs controls and shown adjacent to representative petri dishes. Average values of three experiments ±S.D. (*n* = 3) are shown. ^*^P < 0.05; ^**^P < 0.01; ^***^P < 0.001; difference vs control group, ^#^*P < 0.05;* ^##^*P < 0.01;* ^###^*P < 0.001*; difference vs gemcitabine group. (**F**) BxPC-3, PANC- 1 and MIA-PaCa-2 cells were pre-incubated with 5 μM CPX and/or 10 mM gemcitabine for 4 hours to assess ROS production. Here we show results obtained by OHdG measurements. Absorbance detection was measured using a microplate reader ^*^ *P* < *0.05*, ^**^P < 0.01 vs. control group. ^#^, *P<0.05* vs.CPX group, (Student's *t*-test). All values are expressed as average ±S.D. (*n* = 3). Gemci; Gemcitabine.

Afterwards, we performed a series of clonogenic survival assays to assess the sensitivity of BxPc3, Panc1 and MIA PaCa-2 cells to CPX (5 μΜ) alone or in combination with gemcitabine (10 mM). After 7 days, colonies were counted from each group and then normalized to the control group and represented as a percentage of colonies. Gemcitabine decreased clonogenicity greater in MIA PaCa-2 (47%, *p* < 0.05), than that in PANC-1 (26.92%) and BxPc3 cells (29.8%, *p* < 0.05), versus untreated groups. CPX suppressed clonogenicity much greater than gemcitabine treatment in MIA PaCa-2 (76.2%, *p* < 0.01), PANC-1 (64.1%, *p* < 0.01) and in BxPc3 cells (70.85%, *p* < 0.01). These data provide sufficient information to assess the differences in viability between untreated cells, controls (DMSO) and the cells that have undergone gemcitabine alone and CPX alone treatments. These findings indicate that CPX more efficiently decreased the number of colonies versus gemcitabine. The combination of gemcitabine with CPX had a more robust response to gemcitabine-induced antitumor effect in MIA PaCa-2 (98.1%, *p* < 0.001), than that in PANC-1 (54.28%, *p* < 0.001) and in BxPc3 cells (55.3%, *p* < 0.001), in terms of drug-induced loss of clonogenicity (Figure 1E). Combined exposure to both gemcitabine and CPX more dramatic reduced the survival of the pancreatic cells, indicating that there is synergistic activity between gemcitabine and CPX (Figure 1D, 1E).

### CPX produces excessive ROS levels in comparison with gemcitabine, in a panel of human pancreatic cancer cell lines, *in vitro*

It is well known that reactive oxygen species (ROS) -induces DNA damage. There are evidence showing that high levels of ROS can cause cancer cell death via apoptosis (27). As shown in Figure 2, gemcitabine stimulated the production of ROS in human pancreatic *cell lines BxPC-3*, *PANC-1* and *MIA*-*PaCa*-*2*. CPX treatment significantly (*P* < *0.05*) further stimulated the production of ROS. Gemcitabine and CPX co-culture significantly (*P* < *0.01*) strongly triggered the production of ROS in the three pancreatic cell lines (Figure 1F). Thus, increasing oxidative stress by generating ROS exogenously may be selective for cancer cells without affecting normal cells.

**Figure 2:** CPX decreases protein levels of Bcl-xL and survivin, increases cleavage of Bcl-2 and promotes apoptosis, more efficiently compared to gemcitabine (**A**) BxPC-3, PANC- 1 and MIA-PaCa-2 cells were cultured with 5 μM CPX and/or 10mM gemcitabine for 48 h. The cells were harvested and processed for apoptosis assay using the Annexin V-FITC Apoptosis Detection Kit /PI staining and flow cytometry. The total percent of apoptotic cells are presented of three independent experiments that yielded similar results as mean ± S.D. (*n* = 3). ^*^P < 0.05; ^**^P < 0.01; ^***^P < 0.001, difference versus control group, ^#^*P < 0.05;* ^##^*P < 0.01* difference versus gemcitabine-treated group. Gemci; Gemcitabine. (**B**) BxPC-3, PANC- 1 and MIA-PaCa-2 cells were treated with 5μM CPX and/or 10mM gemcitabine for 24 hours. The cells were harvested and subjected to Western blotting assay. Actin was used as loading control. The densitometric quantification of apoptosis-related protein levels (normalized to the actin levels) are shown adjacent to each immunoblot and reflects average values ± SEM of at least 3 independent experiments. ^*^p < 0.05 ^**^P < 0.01 vs. control group. (**C**) Relative activities of caspases -2,-3,-6,-8,-9 after treatment of BxPC-3, PANC- 1 and MIA-PaCa-2 cells with 5μM CPX and/or 10mM gemcitabine. Average values of three replicate experiments ± S.D. are shown. ^*^P < 0.05; ^**^P < 0.01; ^***^P < 0.001, difference vs control group, ^#^*P < 0.05;* ^##^*P < 0.01;* ^###^*P < 0.001*; difference vs gemcitabine group. (Student's *t*-test).

### CPX enhances gemcitabine induction of pancreatic cancer cell apoptosis

To examine whether the inhibitory effects of CPX were correlated with the gemcitabine induction of pancreatic cancer cell apoptosis, BxPc3, Panc1 and MIA PaCa-2 cells were treated with CPX (5μΜ) and gemcitabine (10mM), alone or in combination for 48 h. Then cells were analyzed by Annexin V-FITC/PI double staining flow cytometry (Figure 2A). CPX treatment showed rise to an apoptotic effect, compared to gemcitabine. Co-treatment of gemcitabine with CPX had notably higher apoptosis rates for BxPc3, Panc1 and MIA PaCa-2 cells compared to the control and gemcitabine groups, respectively (Figure 2A, left and right panels). These results illustrate that CPX significantly contributed to reduce proliferation, demonstrating that CPX has a role in apoptotic cell death by both single-drug therapy and combined drug therapy.

### CPX inhibits Bcl-xL and survivin and increases cleavages of caspase 3 protein levels, resulting in apoptosis

To further elucidate the mechanism by which CPX induces apoptosis of pancreatic tumor cells, we examined the expression of anti-apoptotic proteins (Bcl-xL, survivin and cleaved caspase 3). CPX markedly decreased Bcl-xL and survivin levels, and increased cleavage of caspase 3, indicating caspase-dependent apoptosis. The same trend was observed in the three pancreatic cell lines (Figure 2B). Moreover, both CPX and gemcitabine caused a pronounced decrease in Bcl-XL and survivin protein levels and significant increase in cleaved caspase-3 protein levels compared with gemcitabine monotherapy.

### The activation of caspases was consistently more potent after CPX treatment than after gemcitabine treatment, in human pancreatic cancer cells

In order to examine whether different treatments activate distinct caspases preferentially, BxPc3, Panc1 and MIA PaCa-2 cells were exposed to gemcitabine and CPX, alone or in combination, and the activity of caspases-2,-3,-6,-8,-9 were assessed. As shown in Figure 2C, with the exception of caspase 2, a trend towards an increase in the activity of all caspases was detected in all pancreatic cells for CPX treatment alone and in combination with gemcitabine. Furthermore, caspase-3 showed significant higher activity when CPX was co-treated with gemcitabine (Figure 2C). These data indicate a fundamental role of the above caspases in the CPX mediated gemcitabine reducing effect on human pancreatic cell survival.

### CPX downregulates EGFR signaling compared with gemcitabine, in human pancreatic cell lines

We continued this study by examining the effect of gemcitabine and CPX on EGFR signaling in BxPc3, Panc1 and MIA PaCa-2 cells. These cell lines were treated for 2 hours with gemcitabine alone, CPX alone, or combined. Phosphorylation of EGFR at Tyr1068 was reduced in BxPc3, Panc1 and MIA-PACA-2 cells in response to CPX alone. Furthermore, we found that co-treatment of gemcitabine with CPX blocked the induction of pEGFR in response to gemcitabine. We also examined the levels of phosphorylated AKT (pAKT (S473)) which were also decreased following CPX treatment whereas following gemcitabine treatment, were not affected. In BxPc3, Panc1 and MIA PaCa-2 cells, treatment with CPX or the combination of both, resulted in reduced levels of pAKT (S473). In contrast, pEGFR and pAKT(S473) levels were resistant to gemcitabine alone (Figure 3). CPX can potentially have a fundamental effect on the EGFR signaling network.

**Figure 3:** CPX treatment more down-regulate pEGFR and pAKT (S473) more efficiently in comparison with gemcitabine treatment BxPC-3, PANC- 1 and MIA-PaCa-2 cells were pre-treated for 2 hours with 5 μM CPX and/or 10mM gemcitabine and then were harvested for immunoblotting assay. Actin levels were assessed as a loading control. The intensities of pEGFR (Y1068) /total EGFR and pAKT (S473)/total AKT in gemcitabine (10mM) untreated/treated cells, with/without CPX (5 μΜ) are represented in the graphs which are shown in the lower panel and reflects average values ± SEM of at least 3 independent experiments. ^*^P < 0.05; ^**^P < 0.01; ^***^P < 0.001, difference versus DMSO group. Gemci; Gemcitabine.

### Inhibitory growth effects of CPX on tumor size in a dose- and time-dependent manner in BxPc3, Panc1 and MIA-PACA-2 xenograft mice

Figure 4A shows the inhibitory effects of increasing doses of CPX on tumor growth in BxPc3, Panc1 and MIA-PACA-2 xenograft mice. The CPX-treated groups (5.0 mg/kg, 15 mg/kg and 25 mg/kg) versus control groups (untreated) at indicated time points demonstrated increased inhibition of tumor growth correlated with increasing doses of CPX. Compared to untreated mice, the daily CPX treatment caused a pronounced tumor regression at dose 15mg/kg and higher. During CPX treatment, a maximal reduction was observed on day 30 and no significant repression was seen on days 2 to 22. The highest CPX (25 mg/kg) dose used was based on experiments with CPX on breast cancer [23] and leukemia xenografts [26].

**Figure 4:** Pharmacodynamic analysis of CPX showed suppression of survivin levels in tumor of human pancreatic xenograft mice as well as inhibition of tumor growth, in a concetration- and time-dependent manner Female SCID mice were inoculated subcutaneously with BxPC-3 (3 × 10^6^ cells/mouse) or PANC- 1 (3 × 10^6^ cells/mouse) or MIA PaCa-2 (3 × 10^6^ cells/mouse) tumor cells. When local tumors were established, mice were randomly subdivided into groups after daily single oral gavage of CPX at concentration 5 mg/kg, 15 mg/kg, and 25mg/kg. Tumor tissues were resected on 0, 5th, 15th, 30th day after the daily administration of CPX. Tumor tissues were also resected on day 35^th^ day (5 days after stopping the administration of CPX). (**A**) The tumor volumes within each cell line group were calculated (thrice/per week) after oral gavage of CPX at 5, 15 and 25 mg/kg daily. The mean ± SD (*n* = 6) data on tumor volumes are presented in the indicated graph ^*^Significant difference (*P < 0.05*), ^**^Significant difference (*P < 0.01*) versus controls (untreated) per time point. (**B**) Western blot analysis was followed for detecting survivin protein levels in tumor tissues (upper panel). The densitometric quantification of survivin reflects average values ± SD (*n* = 3) of at least 3 independent experiments. ^*^p < 0.05 ^**^P < 0.01 ^***^P < 0.001 vs. Control group of the indicated time point (lower panel). (**C**) Survivin levels as measured by ELISA after increasing doses of CPX at 5, 15, 25 mg/kg (*n* = 3 per time point). Survivin reflects average values ± SEM of at least 3 independent experiments. ^*^p < 0.05 ^**^P < 0.01 ^***^P < 0.001 vs. Control group of the indicated time point.

### Inhibitory effects of CPX on survivin levels in a dose and time dependent manner in tumors lysates of BxPc3, Panc1 and MIA-PACA xenograft mice

Minden and his research group [25] have reported that one of the biological responses of tumor cells to CPX therapy was the repression of survivin mRNA expression levels. For that reason, we explored the inhibitory effects of CPX treatment by examining survivin protein levels from tumor tissues before, during, and after CPX administration, as a pharmacodynamic marker to confirm biological tumor response. Compared to untreated mice, daily CPX treatment caused a pronounced decrease of survivin at dose 15mg/kg and higher. During treatment, a maximal reduction was observed on day 30 (Figure 4B) and no significant repression was seen on days 2 to 22. Reduced levels of survivin were retained for at least 5 days after stopping CPX treatment. Inhibition of survivin levels was boosted in conjunction with increasing treatment dose and time. The results of the Western blot coincided with that of the Elisa assay (Figure 4C) performed.

### CPX potentiates the anticancer activity of gemcitabine: inhibits subcutaneous tumor xenograft growth and prolongs survival in pancreatic cancer xenograft mouse models

Having shown that CPX enhances gemcitabine activation and efficacy *in vitro*, we next examined *in vivo* the efficacy using BxPc3, Panc1 and MIA PaCa-2 tumor xenograft models in immune-deficient SCID mice. To determine the efficacy of the CPX treatment strategy of gemcitabine-sensitive (MIA PaCa-2, BxPc3) and -resistant tumor models (Panc1), humanized subcutaneous tumor models were established. We investigated whether administration of CPX increases the anti-cancer activity of gemcitabine in tumor-bearing animals. When tumors volumes reached approximately 100 mm^3^, mice were randomized and divided into four sub-groups for each cell line; control (Vehicle) group, gemcitabine treatment group, CPX treatment group and gemcitabine with CPX treatment group. Next, the mice in the CPX treatment group were treated daily by oral garages with CPX (25 mg/kg), mice in the gemcitabine (60 mg/kg) treatment group were treated three times a week with a continuous i.p. perfusion of gemcitabine (60 mg/kg). Both, CPX and gemcitabine, treatment were well tolerated by mice. As shown in Figure 5 (left panel), treatments significantly inhibited tumor growth in the three pancreatic tumor models, with combination therapy showing increased efficacy compared with either CPX or gemcitabine when administered alone. Furthermore, treatment significantly prolonged the survival of the tumor-bearing animals, with combination treatment essentially preventing the death of animals for the duration of the experiment. The median prolongation of survival was 22 days for Panc1, 47 days for MIA PaCa-2, 54 days for BxPc3 xenografts for the vehicle treated group, which was increased to 40 days for Panc1, 65 days for MIA PaCa-2, and 63 days for BxPc3 xenografts for the gemcitabine-treated group (*P* < 0.05), which was further increased to 53 days for Panc1, 78 days for MIA PaCa-2, and 77 days for BxPc3 xenografts for the CPX-treated group (Figure 5, right panel).

**Figure 5:** CPX monotherapy improves the efficacy of gemcitabine monotherapy on the growth of established local pancreatic tumors in BxPC-3 Panc1 and MIA PaCa-2 xenograft models (**A**) SCID mice were implanted with BxPC-3 Panc1 and MIA PaCa-2 cells. When local tumors were established, animals were randomly subdivided into four groups (i) vehicle; (ii) Gemcitabine alone (60 mg/kg); (iii) CPX alone (25 mg/kg); (iv) Combination of gemcitabine (60 mg/kg) and CPX (25mg/kg) of each cancer cell line, respectively. The animals were continuously gavaged with the agents for 90 days as mentioned in the Materials and Methods section. The tumor volume within each treatment group was calculated (thrice/per week) and presented in the indicated graphs. Values are means, *n* = 6–8. ^*^Significant difference (*P < 0.05*), ^**^Significant difference (*P < 0.01*) versus controls. Combination therapy was significantly more potent and the difference reached significance compared with gemcitabine treatment alone after 31 days for MIA PaCa-2 and 35 days for BxPC-3 and 46 days Panc1 (^#^*P <* 0.05 Student's *t*-test). (**B**) The median survival of BxPC-3, Panc1 and MIA PaCa-2 pancreatic tumors in each treatment group was constructed according to the Kaplan-Meier survival curve; *n* = 6 mice in each sub –group. The *P* values (^*^P, 0.05, ^**^P, 0.01 vs the control group) for survival differences were determined applying log-rank testing (GraphPad Prism 4). CTR, vehicle control; Gemci, Gemcitabine; CPX, ciclopirox.

Detection of Ki-67-positive tumor cells was carried out to examine cell proliferation after treatment. As indicated in Figure 6A, at the end (day 30) of the 4 week treatment cycle, the Ki-67 labeling index showed a reduced number of Ki-67-positive tumor cells in CPX –agent alone or combined with a gemcitabine treatment group in comparison to tumor cells from gemcitabine-treated animals, indicating the advantage of the CPX treatment over gemcitabine (Figure 6B).

**Figure 6:** CPX monotherapy reduces cell proliferation levels, decreases pEFGR (Y1068) and pAKT (S473) levels in tumor cells more robustly in comparison with gemcitabine, however, abolishes gemcitabine-induced ROS levels in pancreatic tissues, *in vivo* (**A**) Schematic representation of the experiment protocol; SCID mice bearing subcutaneous BxPC-3 Panc1 and MIA PaCa-2 tumor xenografts, were grouped into four groups, respectively (i) vehicle (*n* = 6); (ii) Gemcitabine alone (60 mg/kg) (*n* = 6); (iii) CPX alone (25 mg/kg) (*n* = 6);; (iv) Combination of gemcitabine (60mg/kg) and CPX (25 mg/kg) (*n* = 6);. (**B**) Representative images of Ki67-positive cells in tumor tissues from BxPC-3 Panc1 and MIA PaCa-2 tumor xenografts, on day 30 after treatment initiation, were assessed by confocal fluorescence microscopy. Red arrows indicate Ki67-positive cells (**C**) Mice were treated as described in Figure 6A. Tumors were harvested on day 30 of treatment for immunoblotting *(three pooled samples per treatment / cell line for the experiment described in (A)* and the indicated total and phosphorylated proteins were estimated by Western blot analysis of three independent experiments with similar results. (**D**) The levels of 8-hydroxy-2’ -deoxyguanosine (8-OHdG0 (arbitrary units, AU) were verified in the pancreatic tissues of BxPc3, Panc1 and MIA PaCa-2 tumor xenograft models, mice, respectively, treated with CPX and/or gemcitabine on day 30 as indicated in Figure 6A. (*n* = 6 per experimental group). ^*^P < 0.05 (Student's *t*-test). All values are expressed as average ± S.D. CTR, vehicle control; Gemci, Gemcitabine; CPX, ciclopirox.

### CPX inhibits EGFR signaling in comparison with gemcitabine *in vivo*

To characterize the molecular phenotype of tumors treated with CPX and gemcitabine, we analyzed EGFR signaling in BxPC-3, PANC-1 and MIA-PACA-2 tumor xenografts at the end (day 30) of the 2 week treatment. Consistent with our *in vitro* findings, we found that phosphorylation of EGFR at Y1068 and AKT (Ser473) was significantly reduced following treatment only with CPX alone on day 30, although the treatment with gemcitabine did not. In addition, the co-administration of CPX with gemcitabine significantly further reduced EGFR (Y1068) and AKT (Ser473) at the 30 days (Figure 6C).

### Treatment with CPX not only does not affect ROS baseline levels but rather abrogates gemcitabine-induced ROS levels in pancreatic tissues, *in vivo*

In view of the ability of CPX to scavenge ROS [30], we evaluated the levels of 8-hydroxy-2’ -deoxyguanosine (8-OHdG) in the pancreas tissue of human pancreatic tumor xenograft models that have been administrated to CPX alone or gemcitabine alone or in combination with CPX (Figure 6A). As shown in Figure 6D gemcitabine single agent caused a strong induction of ROS accumulation significantly (for BxPC-3, PANC-1; *P* < 0.05, for MIA-PACA-2; *P* < 0.01), whereas CPX single agent did not affect ROS accumulation. CPX has shown to alleviate the levels of ROS in the pancreas tissues of mice treated with gemcitabine.

## DISCUSSION

CPX has recently been repositioned as a potential therapeutic agent to treat patients suffering from human acute myelogenous leukemia [27, 26], breast cancer, rhabdomyosarcoma and colon carcinomas [23]. In preclinical studies, the antitumor properties of CPX are depended at least partly to chelation of intracellular iron, resulting in disruption of cell cycle progression [27]. Correspondingly, CPX due to an iron-dependent modification impairs Wnt signaling in malignant cells [20]. These actions offer a mechanistic basis for CPX anti-tumor responses. Given the findings of our experiments, we pinpoint the comparative benefits of CPX over gemcitabine, a standard chemotherapeutic agent and we elucidate potential effects and mechanisms of gemcitabine plus CPX combination in pancreatic cancer models.

Apoptosis is a complex orchestrated process that is tightly regulated by anti-apoptotic proteins, such as Bcl-xL, and survivin. [32–36]. Overexpression of anti-apoptotic Bcl-xL and survivin proteins protect cancer cells from apoptosis [35–37]. Our study shows that CPX sharply decreased protein levels of these proteins. Moreover, the execution phase of the apoptotic process is mediated by caspases, a large evolutionarily conserved family of cysteine proteases [38]. Indeed, CPX-induced apoptosis of pancreatic cells was mediated via a caspase cascade, especially caspase-3. Our results clearly indicated that CPX-treated cells expressed high levels cleavage of procaspase-3 more effective than gemcitabine treated cells. Furthermore, cell viability and clonogenic assays signify that CPX-related suppression in cell proliferation was more potent than gemcitabine-related suppression. This data are consistent with the notion that CPX monotherapy trigger significantly higher apoptosis rate than gemcitabine monotherapy. Moreover, the combination therapy of CPX and gemcitabine significantly down-regulated Bcl-xL and survivin, which induced pancreatic cancer cell apoptosis at an even higher rate of as compared to single-drug treatment.

Increasing evidence support that pancreatic cancer xenograft mouse models imitates the robustly progressive nature of pancreatic cancer [39,40]. Our preclinical pharmacodynamic assays exhibited inhibitory growth actions of CPX on tumor volume in a concentration- and time-dependent manner in BxPc3, Panc-1 and MIA-PACA-2 xenograft mice. Our Western blotting and Elisa assays proved that the survivin levels in the tumors of BxPc3, Panc-1 and MIA-PACA-2 xenograft mice markedly abrogated by CPX administration in a time- and concentration -dependent manner. Another noteworthy finding was that survivin levels remain suppressed after 5 days of discontinuation of CPX treatment. These results suggest that survivin is an effective biological / pharmacodynamic biomarker for demonstrating the antitumor efficacy of CPX.

Herein, our results have revealed that CPX monotherapy was undoubtedly more effective than gemcitabine monotherapy. Combination therapy had obviously higher anti-tumor effect on tumor growth and subsequently prolonged survival rate, indicating a synergistic anti-cancer action compared with single-agent gemcitabine / CPX treatment response. These results were also consistent with the reduced proliferation marker (Ki-67) following CPX versus gemcitabine administration, while their combination exhibited even lower Ki-67 scores in pancreatic tumor cells. Moreover, these *in vivo* studies strongly boost the addition of CPX to gemcitabine. This synergistic strategy may represent new avenues for the treatment of patients with pancreatic cancer. The single - drug therapy as well as the co-administered therapy showed not to correlated with toxicity events, such as weight loss, cachexia symptoms and morphological changes in tissues during necropsy. These results are consistent with a recent phase I clinical trial of CPX in patients with hematological malignancies, in which CPX has been shown to be well tolerated and without toxicity at dose 40 mg/m^2^ once daily [25].

Ciclopirox has been proposed to act as an iron chelator by inhibiting iron-dependent enzymes, causing oxidative toxicity in fungi [23, 41]. Previous studies have demonstrated that CPX induced autophagy (an evolutionarily catabolic process that involves cell degradation of the dysfunctional / unnecessary components of a cell via the lysosomal machinery) through the production of ROS levels [42] in human rhabdomyosarcoma cells [43, 44]. Increasing evidence also support that CPX can trigger cell death via ROS generation, triggering the caspase-dependent mitochondrial cell death network via activation of p38 [42]. Excessive generation of ROS changes mitochondrial morphology and potential. This fact represents a crucial step for cytochrome C release into the cytosol, triggering the cleaved caspase 3 activation [45, 46]. In our study, we noticed induced ROS levels in the CPX-treated group compared with gemcitabine in human pancreatic cancer cells. Also, we have shown *in vitro* that CPX can enhance gemcitabine's cytotoxicity, suggesting that ROS generation destroys malignant cells by CPX-induced apoptosis. Noteworthy the ROS scavenging activity of CPX inhibits the ROS production of the pancreatic tissues, underlying the beneficial properties of CPX in healthy tissues [30]. We further investigated the role of CPX in ROS generation, in mouse pancreatic tissues followed CPX monotherapy, *in vivo*. Of interest, we found that CPX abolished gemcitabine-enhanced ROS generation in pancreatic tissues, *in vivo*. Therefore, these *in vivo* results outline that CPX may be a better candidate because of its less undesired effect (reducing intracellular ROS) than gemcitabine for pancreatic cancer treatment.

Previous studies have reported that EGFR (epidermal growth factor receptor) is a key regulator in tumorigenesis and tumor development mediated by differentiation, apoptosis and DNA damage response [47–49]. Gemcitabine resistance is correlated to overexpression of pEGFR and consequently an over-stimulation of PI3K/AKT signaling network [50]. Our study identified that CPX was capable to decrease EGFR at Y1068 and pAKT (S473) levels in pancreatic cancer cells, which, consecutively, inhibit pancreatic cell growth, by the end of the *in vivo* treatment. These results were consistent with our *in vitro* findings. Moreover, our results *in vitro* showed that, inhibition of EGFR by co-treatment with these drugs further enhanced CPX-induced procaspase-3 and Bcl-2 /survivin downregulation Collectively, these results indicate that CPX-enhances ROS accumulation in pancreatic cancer cells, which results in inhibition of EGFR/AKT signalling and, ultimately, cancer cell death.

In conclusion, our reported data suggest that CPX has profound anti-tumor activity *in vivo* (in murine pancreatic cancer models) and *in vitro* (in a panel of human pancreatic cancer lines). These pre-clinical results also verify a superior efficacy of CPX over gemcitabine alone, while their combination seems to exhibit a synergistic anti-tumor effect. CPX alone or in combination with gemcitabine reduced pEGFR (Y1068) and pAKT (S473) levels through accumulation of ROS to thereby sensitize pancreatic cancer cells to increased apoptosis. These findings provide strong supporting evidence for the anti-tumor activity of CPX and offer the rationale for further clinical testing of CPX plus gemcitabine in patients with locally advanced and/or metastatic pancreatic cancer.

## MATERIALS AND METHODS

### Cell lines

BxPC-3 (ATCC^®^ CRL-1687^™^), Panc-1 (ATCC^®^ CRL-1469^™^), and MIA PaCa-2 (ATCC^®^ CRL-1420^™^), (human pancreatic cancer cell lines) were purchased from American Type Culture Collection (ATCC; Manassas, VA) and sustained in Gibco Gibco DMEM (Panc-1, and MIA PaCa-2) or in RPMI 1640 medium (BxPC-3), with a percentage of 10% fetal bovine serum (FBS) and 100 U/mL of penicillin, and 100 lg/mL of streptomycin solution at 37°C in 5% CO2 in a humidified incubator.

### Drug solutions

CPX (Sigma, St. Louis, MO) was prepared by diluting in 100% ethanol to make a stock solution (100 mM), storage at −20°C. Gemcitabine (Gemzar; provided by Eli Lilly, Indianapolis, IN) was diluted in phosphate-buffered saline (PBS, Gibco BRL) and storage at −20°C.

### 3-(4,5-dimethylthiazol-2-yl)-2,5-diphenyltetrazolium bromide (MTT) cell proliferation assay

BxPC-3, Panc-1, and MIA PaCa-2 cells were reseted in 96-well plates in their respective culture media, at a density of 1 × 10^4^ cells /well (in triplicate) in 100 μL medium. The next day, after starvation, cells were exposed to gemcitabine (0–20 μM) or exposed to CPX (0–20 μM) for 72 h, or exposed to CPX (5 μΜ) in combination with gemcitabine (10 mM) for 72 h. After 72 h, MTT (5 mg/mL) was added to the wells and then 96-well plates were incubated for 4 h. Subsequently, 100 μL DMSO in (dimethyl sulfoxide) was added. Absorbance (OD) was read at 570 nm on a Microplate Reader (BIO-TEK Instruments Inc., Bad Friedrichshall, Germany).

### Apoptosis assay

In brief, cells (6 × 10^5^ cells/well) were seeded in 6-well plates under storage culture conditions overnight at the 37°C humidified incubator with 5% CO2. The next day, the cells were cultured with CPX (5 μM) alone or gemcitabine (10 mM) alone or cultured to CPX (5 μM) in combination with gemcitabine (10 mM) for 48 h. The cells were then trypsinized (Gibco Trypsin-EDTA, Invitrogen), washed and processed for apoptosis assay with the Annexin V-FITC Apoptosis Detection Kit (Thermo Fisher Scientific) in agreement with the instructions of the manufacturer. Cells incubated with vehicle alone (100% ethanol) were utilized as a control.

### Western blot assays

For immunoblot analysis, tumor tissues and human pancreatic cells (BxPC-3, Panc-1, and MIA PaCa-2) were homogenized or lysed, respectively, with ice-cold RIPA buffer (Pierce; Thermo Fisher Scientific, Inc.) supplemented by a protease and phosphatase inhibitor cocktail (Pierce; Thermo Fisher Scientific, Inc.) in agreement with the manufacturer's procedures. The protein fractions were calculated using the Bradford assay (Bio-Rad Laboratories, Hercules, CA). Tissues were homogenized and cell lysates were subjected to SDS-PAGE (sodium dodecyl sulfate–polyacrylamide gel electrophoresis) and then transferred to a sheet of nitrocellulose membranes (Macherey-Nagel, Germany). The blots were blocked with 5% nonfat dried milk and incubated with primary antibodies Cleaved Caspase-3 (#9661), Bcl-xL (#2764), Survivin (#2808), EGF Receptor (D38B1) XP (#4267), Phospho-EGF Receptor (Tyr1068) (#2234), Akt (#4685), Phospho-Akt (Ser473) (#4060), (Cell Signaling Technology, Beverly, MA) and actin, clone C4 MAB1501 (Millipore, Billerica, MA) overnight, at 4°C. Next, membranes were then re-probed with secondary antibodies for 1h at room temperature, followed by incubation with ECL reagent (Amersham Biosciences), and finally exposed to X-ray film (Fuji, Fischer Scientific). The ImageJ platform (NIH) was employed for protein quantification.

### Detection of apoptosis with caspase colorimetric protease assay kit

In brief, 3 × 10^6^ cells were used for each treatment and were lysed by the addition of 50 μl of lysis buffer and incubated the lysate for 10 min on ice. The supernatants were removed by centrifugation at 14 000 *g* for 1 min. 200 μg of the supernatant was mixed with 50 μl of the 2× reaction buffer provided. Where indicated, 5 μl of a 4 mM solution of the appropriate substrate for caspase 2, 3, and 9 was added to each sample and pre-incubated with the indicated specimens at 37°C for 1–2 h. The absorbance was measured at 405 nm microplate reader. Each data point was carried out in triplicate.

### Survival clonogenic assay

For the colony formation assay, cells were seeded in 12-well culture dishes treated with CPX (5 μM) and gemcitabine (10mM) alone or co-added with CPX for 24 h. The cells were then collected and seeded into 100 mm culture plates for 2 weeks. The formed colonies were washed and fixed in prepared fixative [methanol: acetic acid (3:1)] solution and finally stained with hematoxylin (Mayer's).

### Pharmacodynamic analysis based on tumor volume and survivin levels in tumor tissues of BxPC-3, Panc-1, and MIA PaCa-2 xenograft mice

Seven-week-old female SCID mice were purchased from the Jackson Laboratories (Bar Harbor, ME). Animal care and experiments were carried out with the guidelines of the Laboratory Animal Facilities (National and Kapodistrian University of Athens), Medical School Bioethics Committee in agreement with the European Union (approval no. 7924 /12/12/2014). Each group of mice was injected intraperitoneally into the right flank with 2.5 × 10^6^ BxPC-3, Panc-1, and MIA PaCa-2 pancreatic cancer cells, respectively, in 100 μl serum-free respective culture media. The animals were examined for the development of tumors in three dimensions externally, using a digital caliper. Mice were grouped according to their similar tumor volume. The tumor volumes were determined by the formula tumor volume = [(length × width^2^) / 2]. When the average tumor volume per mouse was between 80 and 100 mm^3^, mice were randomly assigned to the following treatment groups: Control group (4% ethanol, 5.2% Tween 80, and 5.2% PEG 400); CPX at 5mg/kg; CPX at 15mg/kg; CPX at 25mg/kg. The drug was administered via oral gavage daily, and the tumor volume was measured every 2 days. Drug administration lasted for 30 days unless the mice died.

Western blotting was employed to explore the inhibitory effect of CPX on survivin levels in the tumors of BxPC-3, Panc-1, and MIA PaCa-2 xenograft mice. Tumor tissues were removed and stored at −20°C for further examination. Western blotting assays were executed as previously described. Also, the survivin amount was measured by human survivin ELISA kits (ab183361) according to manufacturer's instructions. Enzymatic reaction was read at 450 nm on an AutoReader III (Ortho Diagnostic Systems).

### Tumor volume and survival of human xenograft mouse models

Treatment with drugs started when the average tumor volume per mouse was between 80 and 100 mm^3^. Then each group of treated mice was divided into four sub-groups. Mice from each sub-group were treated daily by oral gavage with vehicle control, or CPX (25 mg/kg) prepared in a solution (4% ethanol, 5.2% Tween 80, and 5.2% PEG 400) or with i.p. injections of gemcitabine [60 mg/kg thrice weekly] alone or co-administrated with CPX (25 mg/kg). Tumor volumes were marked until day 90. At the end point of the experiments, mice were sacrificed by cervical dislocation, and tumors and pancreatic tissues were collected for further analysis. For survival analysis, death events were scored; when mice died, or when they became moribund and had to be killed, or when they had to be killed because their tumor exceeded 10% of body weight. The median survival of BxPC-3, Panc1 and MIA PaCa-2 pancreatic tumors in each treatment group was monitored according to the Kaplan-Meier survival curve; n = 6 mice in each sub –group.

### Measurement of ROS production: monitoring 8-OHdG levels

Mice were anesthetized by intraperitoneal injections of Ketamine (100 mg/kg) and Xylazine (16mg/kg) before the performance of surgical procedures. Pancreatic tissues were excised. Next, the tissues were frozen in liquid nitrogen and stored at −80°C until analyzed. Subsequently, for cell cultures and pancreatic tissues, oxidative damage 8-OHdG was quantified with the highly sensitive 8-OHdG check enzyme-linked immunosorbent assay (ELISA) kit (Genox Corp., Baltimore, MD) in agreement with the manufacturer's instructions, as described in [30].

### Immunofluorescence

Frozen tissue sections were fixed in 4% paraformaldehyde. Next, were initially incubated with Ki-67 (D3B5) (#11882), then washed, and afterward incubated with secondary goat anti-rabbit antibody (Invitrogen). Staining for ki67 was conducted on three tumors from each subgroup of mice. Photographs were taken under a confocal microscope (Leica 626 TCS SPE confocal laser scanning microscope).

### Statistical analysis

All experimental results were carried out from at least three independent representative experiments and expressed as mean values ± SD (standard deviation). The results were evaluated by ANOVA (one-way analysis of variance). Statistical significance was inferred when *P* < *0.05*. Statistical analysis to compare differences in survival times across treatment groups was performed using the log-rank test, and differences were reported to be significant when *P* < *0.05*.
